The article "Brain metabolic changes in Hodgkin disease patients following diagnosis and during the disease course: An 18F-FDG PET/CT study" was published in 2014. Journal: Oncol Lett.

# Brain metabolic changes in Hodgkin disease patients following diagnosis and during the disease course: An ^18^F-FDG PET/CT study

**DOI:** 10.3892/ol.2014.2765

**Published:** 2014-12-03

**Authors:** AGOSTINO CHIARAVALLOTI, MARCO PAGANI, MARIA CANTONETTI, BARBARA DI PIETRO, MARIO TAVOLOZZA, LAURA TRAVASCIO, DANIELE DI BIAGIO, ROBERTA DANIELI, ORAZIO SCHILLACI

**Affiliations:** 1 Department of Biomedicine and Prevention, University of Rome Tor Vergata, Rome I-00133, Italy; 2 Institute of Cognitive Sciences and Technologies, The National Research Council, Rome I-00185, Italy; 3 Department of Nuclear Medicine, Karolinska Hospital, Stockholm SE-17176, Sweden; 4 Department of Nuclear Medicine, IRCCS Neuromed, Pozzilli I-86077, Italy

**Keywords:** adriamycin, bleomycin, vinblastine and dacarbazine, chemotherapy, chemobrain, Hodgkin disease, positron emission tomography

## Abstract

The aim of the present study was to investigate brain glucose metabolism in patients with Hodgkin disease (HD) after diagnosis and during chemotherapy treatment. Following the administration of first-line doxorubicin, bleomycin, vinblastine and dacarbazine (ABVD) chemotherapy, 74 HD patients underwent ^18^F-fluoro-2-deoxy-D-glucose (^18^F-FDG) positron emission tomography (PET)/computed tomography brain scans, both baseline (PET0) and interim (PET2) at the Department of Biomedicine and Prevention, University of Rome Tor Vergata (Rome, Italy). Fifty-seven patients were further evaluated 15±6 days after four additional cycles (PET6). Furthermore, a control group (CG) of 40 chemotherapy-naïve subjects was enrolled. Differences in brain ^18^F-FDG uptake between the CG, PET0, PET2 and PET6 scans were analyzed using statistical parametric mapping. Compared with the PET0 and CG scans, the PET2 scan demonstrated a higher metabolic activity in Brodmann area (BA) 39, and a metabolic reduction in BA 11 bilaterally and in left BA 32. All of these changes disappeared at PET6. The results of the present study indicate that ABVD chemotherapy has a limited impact on brain metabolism.

## Introduction

Hodgkin disease (HD) is a lymphoproliferative disorder with an incidence rate of 2.7–2.8 per 100,000 individuals in the UK and the USA in 2013 (1). Doxorubicin, bleomycin, vinblastine and dacarbazine (ABVD) chemotherapy (CHT) is routinely used in the treatment of HD (2), and is less toxic than other chemotherapeutic schemes*,* such as mechlorethamine, vincristine, procarbazine and prednisone (3), and bleomycin, etoposide, doxorubicin, cyclophosphamide, vincristine, procarbazine and prednisone regimens (4).

In a recent study investigating the brain glucose metabolism in HD patients by means of 2-[^18^F] fluoro-2-deoxy-D-glucose (^18^F-FDG) positron emission tomography/computed tomography (PET/CT), the hypothesis of brain damage induced by ABVD CHT treatment was dismissed (5). However, a strong body of evidence demonstrates the coexistence of depression and cancer, with a 20–50% prevalence of depression in patients exhibiting solid tumors (6). Furthermore, various studies report a direct correlation between the rapid progression of cancer and severe depression (7). This is consistent with our previous study, which supports the hypothesis that metabolic changes following CHT may correlate with the transient depressive state of cancer patients after diagnosis, followed by an improvement in general and psychological conditions due to a positive therapeutic response (5).

The aim of the present study was to investigate the impact of ABVD CHT on a larger cohort of HD patients, evaluating the brain metabolic changes during the various steps of CHT and comparing them with an age-matched control group (CG). Furthermore, the possible role of disease severity as a variable affecting the brain metabolic changes was investigated in the HD patients.

## Patients and methods

### Patients and CG

From September 2008 to September 2012, 74 patients (males, 32; females, 42; mean age, 32±11 years) with biopsy-diagnosed HD, who were included in a national study evaluating the early treatment response to ABVD CHT (8), underwent a ^18^F-FDG PET/CT brain scan in 3D mode (9) in association with a whole body staging PET/CT study. According to the Ann Arbor staging Criteria (10), 11, 35, 11 and 17 patients exhibited stages I, II, III and IV HD, respectively.

In accordance with previous studies (11–13), all patients underwent the initial PET/CT scan (PET0) within one week of HD diagnosis. A second PET/CT scan (PET2) was performed in all patients, 15±5 days after the first two ABVD cycles. Written informed consent was obtained for a third brain PET/CT scan (PET6) from 57 patients (females, 31; males, 26; mean age, 31±10 years), which was performed 15±4 days after four additional one-month ABVD cycles, for a total of six cycles.

Forty CHT-naïve subjects (males, 22; females, 18; mean age, 36±7 years) undergoing a ^18^F-FDG PET/CT and found to be completely negative for various diseases were enrolled in the study and served as the CG (14).

Patients and CG subjects with a history of diabetes, other carcinomas, human immunodeficiency virus, neurological, psychiatric or mood disorders, surgery, radiation or trauma to the brain were excluded from the present study. Furthermore, a number of patients treated with agents that could interfere with ^18^F-FDG uptake and distribution in the brain were excluded from the present study (16). No patients demonstrated liver or renal damage, and no patients were pregnant or breastfeeding. Informed consent was obtained from all of the patients, in accordance with the Declaration of Helsinki, and the present study was approved by the ethics committee of the Hospital of Tor Vergata (Rome, Italy).

### Treatment strategy

ABVD cycles were repeated every 28 days. A cycle of treatment consisted of the following on day one: doxorubicin, 25 mg/m^2^; bleomycin, 10,000 units/m^2^; vinblastine, 6 mg/m^2^; and dacarbazine, 375 mg/m^2^, which were administered intravenously (i.v.). The dose intensity was 100%, regardless of patient blood count.

### PET/CT scanning

The Discovery ST16 PET/CT system (GE Medical Systems, Powell, TN, USA) was used to assess ^18^F-FDG distribution in all patients in 3D mode in a 128×128 matrix. Reconstruction was performed using the 3D reconstruction method of ordered subsets expectation maximization with 21 subsets and four iterations. The system combines a high-speed ultra 16-detector-row (912 detectors/row) CT unit and a PET scanner with 10,080 bismuth germanate crystals in 24 rings. The axial full width half maximum (FWHM) was 1 cm (3D mode radius, 5.2 mm) and the axial field-of-view was 157 mm. All patients and CG subjects fasted for a minimum of 5 h prior to i.v. ^18^F-FDG injection to produce a serum glucose level of ≤120 mg/ml. All of the subjects in the present study were intravenously injected with 3 MBq/kg (range, 210–350 MBq) ^18^F-FDG and hydrated with 500 ml i.v. saline NaCl 0.9%.

^18^F-FDG was administered to each patient in a dedicated, dark room. All of the patients were required to remain in a resting condition with closed eyes prior to the PET/CT scan. Following a 45 min rest period, the brain PET/CT scan was performed by placing the patient’s head in a support. A low-amperage CT scan of the head was performed for attenuation correction (40 mA; 120 Kv), prior to obtaining the PET image. The duration of the brain PET image set acquisition was 15 min in all of the patients. All brain PET scans were performed prior to the whole body PET scan, consisting of a low-amperage CT scan for attenuation correction of PET images (80 mA; 140 kV; field of view ~450±5 mm; CT slice thickness, 3.75 mm). The CT Dose Index for ldCT was 4.0175 (±0.84) mGy and the dose-length product was 473.296 (±161.09) mGy-cm. After non-enhanced CT, total-body PET examination in the caudocranial direction from the upper thighs to the vertex was performed (every bed of the PET acquisition lasted 3.5 min). Reconstruction was performed using the 3-dimensional reconstruction method of ordered-subsets expectation maximization (OSEM) with 30 subsets and two iterations.

### Statistical analysis

Differences in brain ^18^F-FDG uptake were analyzed using statistical parametric mapping (SPM2; Wellcome Department of Cognitive Neurology, London, UK) implemented in MATLAB 6.5 (Mathworks, Inc., Natick, MA, USA). PET data were subjected to linear (affine) and non-linear spatial normalization into the Montreal Neurological Institute space. The spatially normalized images were smoothed with a 12-mm isotropic Gaussian filter to blur for individual variations in gyral anatomy and to increase the signal-to-noise ratio. Images were globally normalized to 50 ml/100 ml/min using proportional scaling to remove the confounding effects of changes in the global cerebral glucose consumption, with a masking threshold of 0.8. The resulting statistical parametric maps, SPM{t}, were transformed into normal distribution (SPM{z}) units. SPM coordinates were corrected to match the Talairach coordinates, according to the method implemented by Brett (http://imaging.mrc-cbu.cam.ac.uk/imaging/MniTalairach). Subsequently, Brodmann areas (BAs) were identified at a range of 0 to 3 mm from the corrected Talairach coordinates of the SPM output isocenters, using Talairach Client software (http://www.talairach.org/client.html). Consistent with Bennett *et al* (15), the threshold of the SPM{t} maps was P<0.05, corrected for multiple comparisons using false discovery rate (FDR) at voxel level, and P<0.01, corrected for multiple comparisons using FDR at cluster level. Due to the explorative nature of the present study, when statistically significant differences were not identified at such conservative thresholds, a threshold of P<0.001 uncorrected at voxel level was set. Only those clusters containing >125 contiguous voxels (i.e. >5×5×5 voxels or >11×11×11 mm) were accepted as significant, due to the partial volume effect caused by the poor spatial resolution of the PET camera (~2 × FWHM). The voxel-based analyses were performed using a modality-adjusted paired t-test (two conditions, one scan/condition) and the following comparisons were assessed: i) PET0 vs. PET2 and vice versa; ii) PET0 vs. PET6 and vice versa, CG vs. PET0, CG vs. PET2, CG vs. PET6 and vice versa. Age and gender were used as nuisance variables in all analyses and disease staging was added as nuisance variable in the CG vs. PET2 comparison. Two-way analysis of variance was used in demographic data analyses to assess differences in gender and age. P≤0.05 was considered to indicate a statistically significant difference and, thus, a valid hypothesis.

## Results

No significant differences were identified in age and gender between HD and CG subjects. However, when PET2 data were subtracted from PET0 and CG data, a significant hypometabolic area including a portion of the orbitofrontal cortex (OFC) bilaterally (BA11) and left anterior cingulate cortex (ACC; BA32; Table I) was identified. When compared with PET0 (Table II; Fig. 1) and CG (Fig. 2) scans, PET2 scans demonstrated a significantly higher ^18^F-FDG uptake distribution in the right angular gyrus (BA39; Table I). No significant differences were identified when subtracting PET6 from PET0 and CG scans and vice versa. Furthermore, the ^18^F-FDG uptake distribution changes identified at PET2 disappeared at PET6, and no significant changes were identified between PET6 and PET2, PET0 or CG at any of the explored statistical thresholds.

When using the stage of the disease as the nuisance variable, no significant differences were identified in the comparisons between PET0, PET2 or PET6 data and CG data.

## Discussion

The predominant finding of the present study was a significant hypometabolism in OFC bilaterally (BA11) and in the left ACC (BA32), and an increased glucose consumption in the right parietal cortex, in HD patients following the first two CHT cycles. These changes disappeared at the termination of the therapy, six months after diagnosis.

The present study confirms, in a larger series of patients, the results of a previous report and, thus, reinforces its reliability (5). Furthermore, the present study compared the metabolic status of HD patients with that of a CG, improving the design and the overall statistical power of the study.

Possible CHT-induced damage in BAs 11 and 32 may be important in the reduced brain glucose metabolism in these areas following the first two cycles of CHT. Although chemotherapeutic agents typically have restricted direct access to brain tissue due to the blood-brain barrier, animal studies indicate that even chemotherapeutic agents not known to readily cross the blood-brain barrier (for example, doxorubicin used in the present study) are associated with reduced neurogenesis (16,17). In contrast to the previous study using significantly fewer patients (5), the current study did not demonstrate any differences between the PET6 and PET0 ^18^F-FDG distributions. Furthermore, no significant differences were detected between the CG scan and the brain PET scan at the termination of therapy (PET6).

In the case of CHT-induced brain damage, a diffuse cortical and sub-cortical reduction in brain glucose consumption at PET2, followed by a further reduction after four more CHT cycles, would be expected (18). The present study demonstrated that the metabolic changes that occurred during the disease course and the restoration of normal metabolism in the ACC and PFC at the termination of therapy do not appear to be associated with the total dose of CHT administered.

These findings, in particular those derived from the comparison with CG subjects, are in disagreement with a previously published study exploring functional changes in the brains of CHT-treated patients (19), and dispute claims that ABVD CHT may induce permanent brain damage (19). A previous study evaluating the impact of CHT in female breast cancer patients using magnetic resonance imaging indicated that CHT may cause permanent disruption in the networks of various brain regions (in particular in the hippocampus), thus, directly affecting cerebral function in these areas (20). These disruptions may be associated with specific activation/deactivation patterns in different areas of the cerebral cortical during tasks and at rest (for example, the frontal cortex), as reported by Silverman *et al* (21).

However, a recent study outlined that, during neuropsychological testing, patients who were treated with CHT performed worse than non-cancer control participants. However, CHT-treated patients improved upon their own pre-CHT baseline and performed better than patients treated without CHT, indicating that the majority of long-term cognitive deficits associated with CHT-treated breast cancer patients are generally small in magnitude (22).

The lack of a permanent brain metabolic dysfunction identified in the present study may be due to the different types of CHT used and the different periods of examination during the disease course (~5–10 years in the cited studies; in the acute phase of CHT in the present case) (20,21). ABVD is considered to be less toxic when compared with other CHT schemes (3,4); however, further studies are required to investigate a possible delayed effect of ABVD CHT on brain function and metabolism.

Various changes in the structure and function of the OFC and ACC have been described in different psychiatric conditions. In particular, structural neuroimaging studies have observed a reduction in the gray matter volume of ACC, and left and right OFC among patients with major depressive disorders (23,24). During traumatic exposure in patients exhibiting post-traumatic stress disorder (PTSD), a significant decrease in cerebral blood flow (CBF) has been identified in the ACC and OFC, and a significant increase in CBF has been identified in right parietal regions (25–28). The temporary reduced brain glucose metabolism in the OFC and ACC, and the increased metabolism in the right parietal cortex may be explained by the presence of an acute anxiety status in the present patients. This hypothesis is consistent with the development of depressive symptoms in cancer patients caused by the stress of diagnosis with a life-threatening disease (29). Additionally, cancer diagnosis and treatment are accompanied by a number of acute and chronic stressors that can impact the patient quality of life (29).

In the present study, all patients examined by PET6 were disease-free for a minimum of 12 months and presented a negative whole body PET scan after two ABVD cycles. Thus, treatment with two cycles of ABVD is associated with a high disease-free survival rate in HD patients (10–12). It is possible that the good prognosis in the present series of patients resulted in the disappearance of psychiatric symptoms (time period, 6–12 months), as previously reported in patients affected by cancer (30). However, various functional imaging analyses of patients exhibiting mood disorders identified an increased or a decreased CBF or metabolism in BA 11 and 32, despite the majority of patients exhibiting increased CBF or metabolism at rest (28,31).

The largest regional metabolic differences were identified in the comparison of PET2 with PET0 and CG (Tables I and II). At this point of the disease course (15±5 days after the first two ABVD cycles), a high level of anxiety would be expected, due to: (i) The recent diagnosis (within two months) and (ii) the uncertainty of the therapeutic outcome (12,13). This acute anxiety may impact brain metabolism and blood flow. Although the patient may remain in a state of anxiety associated with the possibility of disease recurrence prior to PET6 examination (13), no significant differences in brain metabolism were identified when comparing PET6 with PET0 and CG scans. This supports the hypothesis of an acute and transient psychiatric condition that affects patients early during the disease course.

The severity of the disease appears to be associated with metabolic changes observed in the brains of HD patients. When the disease stage was used as a nuisance variable in the comparison of PET2 and CG scans, no significant difference was identified, possibly due to the patient’s perception of a more advanced disease stage as a worse prognostic factor. This is supported by a study performed on a large cohort of patients exhibiting different types of cancer; the presence of metastases was associated with an increased number of anxiety symptoms and early disease stage was associated with fewer depressive symptoms (7,32). However, it has been demonstrated that the distribution of ^18^F-FDG uptake in healthy tissues is associated with disease progression in HD (33). Furthermore, various studies have demonstrated that the tumor or treatment-induced inflammation can promote the production of peripheral proinflammatory cytokines. Proinflammatory cytokines activate central nervous system pathways that may induce behavioral and affective symptoms, such as a depressed mood, fatigue, anorexia, impaired concentration, sleep disturbance, enhanced pain sensitivity and reduced activity (29,34–36). Therefore, subsequent studies should include longitudinal neuropsychological, psychiatric and laboratory assessments.

In contrast to previous reports (5), the present study demonstrated no significant metabolic changes in BA 10 (prefrontal cortex) in HD patients receiving ABVD CHT. This discrepancy may explained by the larger number of patients examined in the present study, introducing a higher inter-individual variability and, thus, no significant differences. The previous (5) and present cluster of voxels resulting from the group comparisons were almost superimposable and the reported results predominantly differ in the coordinates of the isocenters determined by SPM. However, in respect to its functional role in major depression and/or PTSD, the prefrontal cortex and orbito-frontal cortex voxel clusters superimpose well (28). Furthermore, stress symptoms in cancer patients have been previously described (30,37,38), and several studies describe diagnosis-associated psychological trauma in cancer patients and survivors, for example acute and chronic PTSD (39,40).

As the design of the present study did not consider the co-occurrence of HD and other psychiatric disorders, the possible occurrence of an acute and transient anxiety status is only speculative. The present study achieved its aim of evaluating alterations in brain metabolism in HD patients during various stages of ABVD CHT treatment and compared with a CG; however, the impact of the psychological status of the patient was only considered post hoc. Thus, the lack of a neuropsychological or psychiatric evaluation following disease diagnosis and during treatment is an evident limitation of the present study.

Another possible limitation of the present study is the use of a CG of subjects with a negative brain PET scan, as opposed to a group of healthy volunteers. However, it is important to note that the CG was specifically set up for the present study, and identical protocol and scanners were used for patients and controls. This is important in neuroimaging studies where the number of potential confounding variables must be minimized. The use of a CG comprising of a sample of individuals with a negative PET is common, due to the high costs associated with obtaining a cohort of volunteers. Furthermore, the stringent exclusion criteria were the same as those applied in previous investigations (41,42). In addition, using a CG comprised of neurologically healthy subjects undergoing PET scans for other reasons prevents healthy individuals being exposed to radiations and makes the protocol feasible for the majority of PET centers, as it reduces the costs and efforts required to build up CGs comprised of healthy subjects (43).

In conclusion, brain metabolic changes in a large cohort of HD patients during the initial phases of CHT are transient and may be due to an acute anxiety state following disease diagnosis and treatment outcome uncertainty. Further studies integrating this data with neuropsychological, psychiatric and laboratory assessments are necessary to confirm the hypotheses of the present study.

## Figures and Tables

**Figure 1:** Brain 2-[18F] fluoro-2-deoxy-D-glucose positron emission tomography (PET)/computed tomography scan (A) within one week of Hodgkin disease diagnosis (PET0) and (B) 15±5 days after the first two adriamycin, bleomycin, vinblastine and dacarbazine cycles (PET2).

**Figure 2:** (A) Significant cortical hypometabolism in positron emission tomography (PET)2 when compared with the PET0 group. Threshold of P<0.05, corrected for multiple comparisons with false discovery rate at voxel level. (B) High 2-[18F] fluoro-2-deoxy-D-glucose uptake in the right superior parietal lobule in PET2 compared with PET0. Threshold of P<0.001, not corrected for multiple comparisons at voxel level. Coordinate and regional details are presented in Table I. PET0, brain 2-[18F] fluoro-2-deoxy-D-glucose (^18^F-FDG) PET/computed tomography (CT) scan within one week of Hodgkin disease diagnosis; PET2, brain ^18^F-FDG PET/CT scan 15±5 days after the first two adriamycin, bleomycin, vinblastine and dacarbazine cycles.

**Table I:** Statistical parametric mapping comparisons between ^18^F-FDG uptake in PET2 and CG.

	Cluster level			Voxel level			
		
Comparison	Cluster extent	Corrected P-value	Cortical lobe	Talairach coordinates	Maximum Z score	Cortical region	BA
CG-PET2	1729	0.036	L limbic	−4, 43, 7	4.16	Anterior cingulate cortex	32
			L frontal	−13, 48, 22	3.29	Superior frontal gyrus	11
PET2-CG	546	0.048	R parietal	48, −71, 33	4.78	Angular gyrus	39

For each significant cluster, the number of voxels, the corrected P-value and the cortical lobe where the voxel is located are reported at the cluster level; and the coordinates of the Talairach correlation sites, the Z-score of the maximum correlation point, and the corresponding cortical region and BA are reported at the voxel level. When the maximum correlation is achieved outside of the gray matter, the gray matter (BA) in the closest proximity was identified (range, 0–3 mm). Thresholds of P<0.05, corrected for multiple comparisons using the false discovery rate, and P<0.001 uncorrected at voxel level, were implemented for PET2 and CG comparisons.. L, left; R, right; BA, Brodmann’s area.

**Table II:** Statistical parametric mapping comparisons between ^18^F-FDG uptake in PET0 and PET2.

	Cluster level			Voxel level			
		
Comparison	Cluster extent	Corrected P-value	Cortical lobe	Talairach coordinates	Maximum Z score	Cortical region	BA
PET0-PET2	1450	0.017^a^	L limbic	−4, 44, 6	4.21	Anterior cingulate cortex	32
			R frontal	4, 52, −12	3.64	Medial frontal gyrus	11
			L frontal	−8, 48, −26	3.49	Orbital gyrus	11
			L frontal	−14, 48, −24	3.47	Superior frontal gyrus	11
PET2-PET0	844	0.042^a^	R parietal	48, −72, 34	4.55	Angular gyrus	39

For each significant cluster, the number of voxels, the corrected P-value and the cortical lobe where the voxel is located are reported at the cluster level; and the coordinates of the Talairach correlation sites, the Z-score of the maximum correlation point, and the corresponding cortical region and BA are reported at the voxel level. When the maximum correlation is achieved outside of the gray matter, the gray matter (BA) in the closest proximity was identified (range, 0–3 mm). Thresholds of P<0.05, corrected for multiple comparisons using the false discovery rate, and P<0.001 uncorrected at voxel level, were implemented for PET0-PET2 and PET2-PET0 comparisons.

a P<0.05 corrected for multiple comparisons at cluster level.

^18^F-FDG, 2-[18F] fluoro-2-deoxy-D-glucose; PET, positron emission tomography; CT, computed tomography; PET0, brain ^18^F-FDG PET/CT scan within one week of Hodgkin disease diagnosis; PET2, brain ^18^F-FDG PET/CT scan 15±5 days after the first two adriamycin, bleomycin, vinblastine and dacarbazine cycles; CG, control group; BA, Brodmann area; L, left; R, right.
